The article "Uncovering the Key Targets and Therapeutic Mechanisms of Qizhen Capsule in Gastric Cancer through Network Pharmacology and Bioinformatic Analyses" was published in 2022. Journal: Comput Math Methods Med.

# Uncovering the Key Targets and Therapeutic Mechanisms of Qizhen Capsule in Gastric Cancer through Network Pharmacology and Bioinformatic Analyses

**DOI:** 10.1155/2022/1718143

**Published:** 2022-11-10

**Authors:** Wanmei Zhou, Xuefei Yu, Ziwei Zhang, Xiao Wang, Chengdong Nie, Guang Zhang, Ning Chen, Wei Zheng

**Affiliations:** ^1^Harbin University of Commerce, School of Pharmacy, No. 138, Tongda Street, Daoli District, 150076 Harbin, China; ^2^Harbin University of Commerce, School of Library, No. 1, Xuehai Street, Songbei District, 150028 Harbin, China; ^3^Harbin University of Commerce, School of Food Engineering, No. 1, Xuehai Street, Songbei District, 150028 Harbin, China

## Abstract

*Objective*. This study is aimed at screening out effective active compounds of Qizhen capsule (QZC) and exploring the underlying mechanisms against gastric cancer (GACA) by combining both bioinformatic analysis and experimental approaches. Weighted gene coexpression network analysis (WGCNA), network pharmacology, molecular docking simulation, survival analysis, and data-based differential gene and protein expression analysis were employed to predict QZC's potential targets and explore the underlying mechanisms. Subsequently, multiple experiments, including cell viability, apoptosis, and protein expression analyses, were conducted to validate the bioinformatics-predicted therapeutic targets. The results indicated that luteolin, rutin, quercetin, and kaempferol were vital active compounds, and TP53, MAPK1, and AKT1 were key targets. Molecular docking simulation showed that the four abovementioned active compounds had high binding affinities to the three main targets. Enrichment analysis showed that vital active compounds exerted therapeutic effects on GACA through regulating the TP53 pathway, MAPK pathway, and PI3K/AKT pathway. Furthermore, data-based gene expression analysis revealed that TP53 and JUN genes were not only differentially expressed between normal and GACA tissues but also correlated with clinical stages. In parallel, *in vitro* experimental results suggested that QZC exerted therapeutic effects on GACA by decreasing IC_50_ values, downregulating AKT expression, upregulating TP53 and MAPK expression, and increasing apoptosis of SGC-7901 cells. This study highlights the potential candidate biomarkers, therapeutic targets, and basic mechanisms of QZC in treating GACA, providing a foundation for new drug development, target mining, and related animal studies in GACA.

## 1. Introduction

Gastric cancer (GACA), a type of severe fatal disease, continues to be the world's most common and deadly cancer, affecting the health of people, especially the elders. It is the fifth most common cancer and the third leading cause of cancer-related death worldwide, with a high mortality rate of up to 75% and an estimated 783,000 deaths in 2018 [1]. Each year, more than 1 million people are diagnosed with GACA [2]. Therefore, the prevention and treatment of GACA have become a research hotspot. Surgical resection is commonly adopted for GACA patients in early stages, which brings health back to patients to some extent. Nevertheless, for patients with advanced GACA, surgical resection does not show significant effects, with only about 20% of patients surviving 5 years after surgery [3]. As a result, chemotherapy and combination treatments are used as alternative remedial approaches to save the lives of patients with advanced GACA [4]. However, chemotherapy is often accompanied by bone marrow suppression, digestive tract reaction, and other adverse effects, causing poor physical condition, lower immune function, and severe clinical symptoms in patients [3]. For these reasons, GACA patients are unlikely to successfully complete the full course of standardized chemotherapy.

The article "Uncovering the Key Targets and Therapeutic Mechanisms of Qizhen Capsule in Gastric Cancer through Network Pharmacology and Bioinformatic Analyses" was published in 2022. Journal: Comput Math Methods Med.

Traditional Chinese medicine (TCM) is of great importance in fighting against cancer; its excellent curative effects have attracted increasing attentions worldwide [4]. Qizhen capsule (QZC), a mixture of medical herbs including Astragali Radix (AR), Notoginseng Radix Rhizoma (NRER), Isatidis Folium (IF), Paridis Rhizoma (PR), and Margarita (MARG), has been commonly used for treating various cancers, including liver cancer, breast cancer, and gastric cancer, for more than two decades [5]. Furthermore, relative studies have proved that QZC can promote blood circulation to dispel blood stasis and clear away heat and toxic materials. Previous studies suggested that combination of QZC with chemotherapy in treating GACA could reduce drug toxicity and increase drug safety at the same time [6]. In recent years, there are only few reports describing QZC's mechanism against GACA. Moreover, existing studies on the mechanism of QZC against GACA have used a single analytical approach, and there is no systematic description of QZC's pharmacological mechanism and its mechanism of action. The research method used for the mechanism study of QZC against GACA is relatively simple; therefore, the underlying mechanism and effective targets of QZC cannot be described systematically [5, 6]. In addition, the underlying mechanisms of QZC against GACA are still not clear because there are multiple active compounds presented in QZC that might have complicated interactions with different targets.

Weighted gene coexpression network analysis (WGCNA) is a functional bioinformatic method used to identify gene modules for therapeutic targets based on gene coexpression analysis. By systematically analyzing the correlation between modules and clinical features, the modules that are closely associated with clinical characteristics can be proposed, and genes that may exhibit critical functions can be predicted [7]. Network pharmacology is a tool that can be used to explain the foundation of complex biological systems from a network perspective. It can also be used to study molecular mechanisms by which herbal medicines fight against diseases and to construct drug-compound-disease networks. It is systematic, relevant, and predictable [8]. Molecular docking is a method for predicting binding interactions between small molecule ligands and target proteins, and it can also be used to validate targets predicted by network pharmacology. In addition, computer techniques related to molecular docking, such as molecular force field/Poisson Boltzmann surface area model (MM/PBSA), molecular mechanics/generalized Born surface area model (MM/GBSA), and molecular dynamics simulation, have been widely used for screening of key protein inhibitors or agonists in TCM [9–11].

The article "Uncovering the Key Targets and Therapeutic Mechanisms of Qizhen Capsule in Gastric Cancer through Network Pharmacology and Bioinformatic Analyses" was published in 2022. Journal: Comput Math Methods Med.

In this study, we employed both bioinformatic analyses (WGCNA, network pharmacology, molecular docking simulation, survival analysis, and data-based gene and protein expression analysis) and *in vitro* experimental validations (cell viability, apoptosis, and protein expression assay) to investigate the molecular mechanisms of QZC against GACA. The results of this study will deepen our understanding of the molecular mechanisms of QZC against GACA and provide useful information for the diagnosis, treatment, and prognosis of GACA. A flowchart of the technical strategy is shown in Figure 1.

## 2. Materials and Methods

### 2.1. Sample Selections and Preparation of Transcriptome Profiles

GACA RNA sequencing data (*n* = 404) were downloaded from TCGA data portal (https://portal.gdc.cancer.gov/) in January 2021. To get valuable information, the clinical metadata from 404 samples were screened. A total of 67 samples with incomplete data were excluded, and the remaining 337 samples were included for further analysis. Consequently, a total of 15,073 genes that were differently expressed between gastric cancer samples were subjected to WGCNA to identify key modules that were closely associated with GACA.

### 2.2. Weighted Gene Coexpression Network Analysis and Key Module Prediction

The WGCNA package was adopted to construct gene coexpression networks. Based on pairwise Pearson correlation coefficient matrices, a similarity matrix was constructed. Subsequently, the correlation coefficients were calculated by distance correlation. As distance correlation coefficients are always positive, they define an unsigned network in which positive and negative correlations are treated equally. With a power adjacency function, an adjacency matrix was obtained from the similarity matrix. The integration function (pickSoftThreshold) was utilized to select an appropriate soft threshold power *β*. A power of *β* = 2 was chosen as the soft-cutoff parameter. The coexpression similarity was improved to obtain a scale-free topology using the soft threshold function. Subsequently, the topological overlap matrix was reconstructed by evaluating the topological overlap measure (TOM). The TOM similarity was used to derive two useful metrics of weights and distances. The dynamic tree-cut algorithm was employed to pinpoint the gene coexpression module with minModuleSize of 50 and mergeCutHeight of 0.01 [12]. Module eigengene (ME) is an important component for each gene module that represents the overall level of gene expression. Module membership (MM) represents the correlation and the gene expression profile. Gene significance (GS) is the absolute value of the association between a specific gene and a clinical trait. Based on ME, MM, and GS, we were able to correlate various modules to clinical traits and identify critical modules in clinical practice [13]. In addition, other parameters used for analysis were set to the default parameters of the WGCNA package.

The article "Uncovering the Key Targets and Therapeutic Mechanisms of Qizhen Capsule in Gastric Cancer through Network Pharmacology and Bioinformatic Analyses" was published in 2022. Journal: Comput Math Methods Med.

### 2.3. Collection of QZC Compounds and Prediction of Their Targets

By combining various databases as well as biomedical literatures, biomolecular networks can be constructed for a compound [14]. The chemical compounds of QZC were collected from both authoritative databases (TCMSP (https://tcmspw.com/), ETCM (https://www.tcmip.cn/), and TCMID (https://119.3.41.228:8000/tcmid/)) [15] and literatures [16–33]. We used oral bioavailability (OB) and drug-likeness (DL) as indicators to select compounds, and compounds with OB ≥ 30% and DL ≥ 0.18 were selected for further study [34]. In addition, several compounds, such as palmitic acid and ononin, which did not meet the above criteria were also selected for further analysis due to their strong pharmacological activities. Compounds' SMILES files from PubChem (https://pubchem.ncbi.nlm.nih.gov/) were uploaded to the TargetNet webserver (http://targetnet.scbdd.com) and Swiss Target Prediction database (http://www.swisstargetprediction.ch/). Protein targets with a prediction score > 0.9 were retained. Targets of compounds documented in TCMSP were also collected. Predicted protein target information including name and UniProt ID was obtained from the UniProt database (https://www.uniprot.org/). Only human targets were retained for the following analysis.

The article "Uncovering the Key Targets and Therapeutic Mechanisms of Qizhen Capsule in Gastric Cancer through Network Pharmacology and Bioinformatic Analyses" was published in 2022. Journal: Comput Math Methods Med.

### 2.4. Construction of Compound-Target Network

The predicted target information of bioactive compounds and the related information were introduced into Cytoscape 3.8.0 to establish a compound-target network [35]. Nodes represent active compounds or predicted targets, while edges show the interplay between the compounds or predicted targets [36].

### 2.5. Construction of Protein-Protein Interaction (PPI) Network

Search Tool for the Retrieval of Interacting Genes/Proteins (STRING) 10.5 (https://string-db.org/) is a robust algorithm that provides not only known and predicted protein interactions but also direct and indirect protein relationships [37]. Genes overlapping compound-predicted targets and WGCNA significant module targets were introduced into STRING 10.5 for further analysis. The species was set to “*Homo sapiens*,” and a confidence interaction score of 0.9 was chosen [38]. The data were then put into Cytoscape 3.8.0 to establish a PPI network, and the “Network Analyzer” plugin was used to calculate the network's topological parameters.

### 2.6. Enrichment Analysis of Gene Ontology Functional Enrichment (GO) Terms and Kyoto Encyclopedia of Genes and Genomes (KEGG) Pathways

GO functional enrichment and KEGG pathway analysis were performed using the David v6.7 database (https://david.ncifcrf.gov/) to elucidate the role of targets in gene function and signaling pathways. The species was set to “*Homo sapiens*.” *P* ≤ 0.05 were considered statistically significant. GO functional enrichment classified genes into three categories, including cellular component (CC), molecular function (MF), and biological process (BP). According to the results of KEGG analysis, Cytoscape 3.8.0 was used to set up a “target-pathway” network to show potential targets and pathways that were involved in QZC against GACA.

### 2.7. Pathways in Cancer

Selected target genes were introduced into KEGG Mapper (https://www.kegg.jp/kegg/tool/map_pathway2.html) to screen out target genes that were involved in pathways related to cancer.

### 2.8. Molecular Docking Simulation

Molecular docking simulation can be utilized to assess the interaction between ligands and receptors based on geometric complementarity, energy complementarity, and chemical environmental complementarity [39]. The 3D structured PDB files of TP53, EP300, AKT1, MAPK1, SRC, RELA, JUN, and HSP90AA1 were downloaded from the PDB database (https://www.rcsb.org/) [40], processed by AutoDock Tools to get rid of ligands from proteins and nonprotein molecules, and saved as PDB files. The 2D structured SDF files of the key active compounds of QZC were collected from the PubChem database [41]. Subsequently, PyRx software was adopted to upload dehydrated protein files and compound files, which were converted to pdbqt format files [42]. Eventually, AutoDock Vina was used for molecular docking.

The article "Uncovering the Key Targets and Therapeutic Mechanisms of Qizhen Capsule in Gastric Cancer through Network Pharmacology and Bioinformatic Analyses" was published in 2022. Journal: Comput Math Methods Med.

### 2.9. Survival Analysis of PPI Genes

Kaplan-Meier Plotter (http://kmplot.com/analysis/) is an online tool that was used to perform survival analysis of the top eight PPI genes in GACA patients [43]. Recurrence-free survival (RFS) refers to the recurrence-free period of GACA patients, and overall survival (OS) is the time from diagnosis to death. Kaplan-Meier Plotter's chi-squared test was used to identify the relationship between the top eight PPI genes and GACA patients' survival (i.e., RFS or OS) [44]. *P* < 0.05 indicated the genes were associated with survival of GACA patients.

### 2.10. Exploration of PPI Gene Expression and Their Corresponding Protein Expression

The mRNA sequencing data of 443 GACA patients were downloaded from TCGA database (http://cbioportal.org). After deleting samples with incomplete data, a total of 407 samples including 32 normal samples and 375 GACA samples were included. Subsequently, we analyzed the difference in expression levels of the top eight PPI genes between normal and GACA tissues, as well as in the four clinical stages. *P* < 0.05 were considered to be statistically significant [36]. In addition, different protein expression levels were also compared between normal and GACA tissues based on the data acquired from the Human Protein Atlas (HPA) database (https://www.proteinatlas.org/).

### 2.11. Cell Culture and Cell Viability Assay

A CCK-8 kit (Beyotime, Shanghai, China) was adopted to assess the effects of luteolin, rutin, quercetin, or kaempferol on the proliferation of SGC-7901 cells (Shanghai Institute Cell Bank, Chinese Academy of Science). SGC-7901 cells were seeded into 96-well plates (Suyan Biotech, Guangzhou, China) at a density of 1 × 10^4^ cells/100 *μ*L and incubated in the incubator for 24 h. Then, SGC-7901 cells were treated with different concentrations of luteolin, rutin, quercetin, and kaempferol for 24, 48, or 72 h, respectively. Subsequently, SGC-7901 cells were incubated with 100 *μ*L of CCK-8 solution (Beyotime, Shanghai, China) for 2 h. The optical density (OD) at 450 nm was measured using a microplate reader (Ruiyu Biotech, Shanghai, China). The 50% inhibitory concentration (IC_50_) values were calculated using GraphPad Prism 8.0 software.

### 2.12. Apoptosis Assay

SGC-7901 cells in the logarithmic growth phase treated by luteolin, rutin, quercetin, and kaempferol were collected and seeded into 96-well plates (Suyan Biotech, Guangzhou, China) at a density of 5 × 10^4^ cells/mL, followed by incubation overnight at 37°C with 5% CO_2_. SGC-7901 cells were treated with RSM for 24 h and then collected by trypsinization. The treated cells were washed with cold PBS (AR-0192, Boster) and then centrifuged. Finally, we treated them with Annexin V-FITC (C1062M, Beyotime, Shanghai, China) and propidium iodide (PI) at 37°C for 40 min in the dark. SGC-7901 cells were then placed in a water bath under light-proof conditions. The cell circle was analyzed with a flow cytometer (BD FACSCalibur, BD Biosciences, America).

The article "Uncovering the Key Targets and Therapeutic Mechanisms of Qizhen Capsule in Gastric Cancer through Network Pharmacology and Bioinformatic Analyses" was published in 2022. Journal: Comput Math Methods Med.

### 2.13. Western Blot Assay

SGC-7901 cells were lysed with 200 *μ*L of preformulated cell lysis mix (cell lysis solution : protease inhibitor : phosphatase inhibitor = 98 : 1 : 1) for 15 min and then transferred to new 1.5 mL EP tubes. After centrifuging at 12,000 r/min for 15 min, the supernatant was collected. Protein concentration was determined using a BCA Protein Assay Kit (P0012S, Beyotime). Protein separation was achieved by sodium dodecyl sulfate polyacrylamide gel electrophoresis (SDS-PAGE), and resolved proteins were transferred onto a PVDF membrane (Bio-Rad, America). After sealing with 5% skim milk (XB-BD-200, XBSW, Guangzhou, China) at room temperature for 2 h, the protein-containing PVDF membrane was washed with TBST solution. Primary antibodies against p-AKT (Ser473, Affinity), AKT (AF6261, Affinity), p-P53 (9286T, Cell Signaling Technology), P53 (2524S, Cell Signaling Technology), p-MAPK (AF5887, Beyotime, Shanghai, China), MAPK (8690S, Cell Signaling Technology), or GAPDH (endogenous reference) were added, respectively, and incubated overnight at 4°C. After washing the membrane, corresponding secondary antibodies were added and incubated for 1 h at room temperature, and an ECL kit was used for visualization. The gray values for each protein band were recorded using a fully automated chemiluminescence image analyzer. GAPDH was used as an internal reference to calculate the relative expression change of each protein. The protein's gray values were calculated by ImageJ and presented using a bar graph.

### 2.14. Statistical Analysis

All data were shown as the mean ± SD. GraphPad Prism 8.0 software was used to analyze experimental results. Student's *t*-tests were performed to compare quantitative data between groups. *P* < 0.05 was defined as statistically significant.

## 3. Results

### 3.1. Construction of WGCNA Module

In this study, a total of 337 samples and 15,073 genes were selected from TCGA data after normalization for WGCNA. To ensure a scale-free network, a power of *β* = 2 (scale-free *R*^2^ = 0.9) was chosen as the soft-cutoff parameter (Figure 2). Nine modules were identified through average linkage hierarchical clustering (Figure 3).

The article "Uncovering the Key Targets and Therapeutic Mechanisms of Qizhen Capsule in Gastric Cancer through Network Pharmacology and Bioinformatic Analyses" was published in 2022. Journal: Comput Math Methods Med.

### 3.2. Screening of WGCNA Hub Module

Expression levels of the whole module were represented as ME. The relationships between ME and clinical characteristics were evaluated by Pearson's test [45]. *P* < 0.05 was considered statistically significant. Data showed that modules and clinical characteristics were significantly correlated. Based on the association between modules and clinical characteristics (futime, fustat, age, gender, grade, stage, pathologic T, pathologic M, pathologic N, and histological), blue and turquoise modules were predicted to be key modules (Figure 4). Each module consisted of coexpressed RNAs with a high TOM. Genes that were categorized into the same module formed networks and were predicted to participate in analogous biological processes. The networks for key modules were filtered at a weight cutoff of 0.1 between genes. In total, 1,392 or 11,362 genes were acquired for the blue module or turquoise module, respectively.

### 3.3. Screening of Active Compounds of QZC and Their Targets

Chemical compounds of QZC were retrieved in two ways. Some were retrieved from the TCMSP, ETCM, and TCMID; others were collected from literatures. A total of 134 compounds were obtained. Then, compounds obtained from the three databases were screened with the criteria of OB ≥ 30% and DL ≥ 0.18. For compounds obtained from literatures, they were further reviewed, and those without significant anticancer effect were removed. As a result, a total of 35 compounds in AR, 34 compounds in NRER, 16 compounds in IF, 17 compounds in PR, and 3 compounds in MARG were included. Based on compound target collection and prediction, 290 targets from AR, 324 targets from NRER, 159 targets from IF, 207 targets from PR, and 27 targets from MARG were acquired, respectively. In total, 94 compounds and 471 targets were finally retrieved after eliminating duplicates. Detailed information on compounds is listed in Table 1.

### 3.4. Construction and Analysis of Drug-Compound-Target Network

To build a visual active target network, 94 active compounds and 471 target genes were introduced into Cytoscape 3.8.0, which generated 573 nodes (94 active compound nodes, 471 target nodes, and 5 herb nodes) and 2,328 lines (Figure 5). The five orange arrows represented 5 herb nodes; blue circles represented the 471 target notes. Targets with the highest degree values were at the center; green squares represented the 99 active compound nodes, and pink squares represented the active compound nodes with the highest degree values. The nine active component nodes with the highest “degree” values were luteolin, palmitic acid, DL-glucuronic acid, daidzein, rutin, kaempferol, oleic acid, beta-sitosterol, and quercetin. The drug-compound-target network clearly indicated that each active compound had multiple targets, and each target was regulated by several active compounds. These results demonstrated that QZC could exert considerable biological and pharmacological effects through multiple active compounds by binding to different targets.

The article "Uncovering the Key Targets and Therapeutic Mechanisms of Qizhen Capsule in Gastric Cancer through Network Pharmacology and Bioinformatic Analyses" was published in 2022. Journal: Comput Math Methods Med.

### 3.5. Screening of Overlapping Targets and Construction of PPI Network

To optimize gene ranges that might be highly related to QZC's active compounds, we screened target genes overlapping blue module, turquoise module, and compound targets by Venn. A total of 314 overlapping target genes were considered potential targets for QZC against GACA (Figure 6(a)). Next, the STRING database was used to construct a PPI network for these 314 overlapping targets to reveal underlying mechanisms. As shown in Figure 6(b), after removing free genes, 211 nodes and 1,215 linkages between genes were included in potential PPI networks after setting the combined score of 0.9 as the threshold and species as “*Homo sapiens*.” Among them, 24 nodes with BC values > the mean of 0.0173, CC values > the mean of 0.3677, and degree values > the double of 18.692 were defined as the major nodes. And these 24 nodes were predicted to be the potential targets for QZC treating GACA, which included *TP53*, *EP300*, *AKT1*, *MAPK1*, *SRC*, *RELA*, *JUN*, *HSP90AA1*, *MAPK8*, *RHOA*, *MAPK14*, *ESR1*, *NR3C1*, *CDK1*, *EGFR*, *RB1*, *CCND1*, *RXRA*, *CXCL8*, *EDN1*, *PRKCA*, *VEGFA*, *FOS*, and *PRKACA*.

### 3.6. GO Term and KEGG Pathway Enrichment Analysis for Potential Targets

Next, GO enrichment analyses, including biological process (BP), molecular function (MF), and cellular component (CC), were performed to explore the underlying mechanisms of QZC against GACA. In addition, KEGG functional enrichment analysis was also used to gain insights into the mechanisms of QZC in treating GACA. A total of 1,425 GO terms were obtained from GO enrichment analysis of 24 potential target genes, of which 1,230, 107, and 88 terms were from BP, MF, and CC, respectively. The top 10 highly enriched terms for BP, MF, and CC are shown in Figure 7. Moreover, there were 84 entries with FDR < 0.01 and *P* < 0.01 after KEGG enrichment analysis. The findings suggested that QZC might exert its effects through the abovementioned pathways in treating GACA. The top 30 KEGG pathways and their correlations with targets are displayed in Figures 8 and 9, respectively. Among them, 24 targets were significantly enriched in 10 pathways that were closely associated with GACA. Moreover, the most overrepresented signal transduction pathways were PI3K/AKT and MAPK pathways, as shown in Figure 10. These pathways were involved in tumor occurrence and survival which have been demonstrated by many studies and supposed to be key pathways [46–48]. Our results indicated that these pathways and their related targets needed to be further investigated in the mechanistic study of QZC against GACA.

The article "Uncovering the Key Targets and Therapeutic Mechanisms of Qizhen Capsule in Gastric Cancer through Network Pharmacology and Bioinformatic Analyses" was published in 2022. Journal: Comput Math Methods Med.

### 3.7. Molecular Docking Analysis

After network analysis, 8 PPI targets (i.e., TP53, EP300, AKT1, MAPK1, SRC, RELA, JUN, and HSP90AA1) were selected to analyze their molecular docking with 9 highly related QZC compounds (i.e., luteolin, palmitic acid, DL-glucuronic acid, daidzein, rutin, kaempferol, oleic acid, beta-sitosterol, and quercetin) using AutoDock Vina. The docking scores of 8 PPI targets with 9 highly related QZC compounds were shown as a heat map (Figure 11). Binding energy ≤ −5.0 kJ mol^−1^ was used as the key criterion [49]. The binding affinity between targets and active ingredients was better when binding energy was lower [50]. A total of 63 compound-target pairs satisfied the requirements. Of them, ten compound-target pairs with strong binding efficiency are depicted in Figure 12. The maximum binding energy was found in SRC-rutin pairs, forming 8 hydrogen bonds (ARG156, ARG160, GLU159, GLN362, GLU517, TYR519, and PHE520), two hydrophobic bonds (VAL364 and PHE520), *π*-stacking (PHE520), *π*-cation interactions (ARG156), and salt bridges (ARG156, ARG160). In conjunction with literature analysis, the kinase structural domain of SRC is usually located in a docking groove directly below the active site cleft to bind substrates or inhibitory fragments, such as VAL364 and PHE520, which can be linked to kinases via hydrophobic interactions [51, 52]. Note that the N-terminal lobe of the kinase contains a long narrow hydrophobic patch along with the SH2-kinase linker. This is, in part, compensated by ARG156, GLU159, and ARG160 of the A-helix on the C-terminal lobe of the SH2 domain [53, 54]. These sites can be targeted by small molecule inhibitors to form protein-protein interactions through linkages such as hydrogen bonds, *π*-cation interactions, and salt bridges [55]. GLN362 is the terminal core site of the SH3 domain in kinases and can bind targets by means of hydrogen bonds. Studies have shown that mutational activation of pp60c-src could lead to a tumorigenic phenotype in a hamster embryo cell line [56]. Its mutation might have a relationship with tumor development. Yaciuk et al. have compared the effects of carboxyl terminal truncation and point mutations on pp^60c-src^ activities. S-fold-enhanced kinase activity has been measured using the pp^60c-src^ truncation mutant, and translation was found to be terminated after Glu 517 [57]. Other studies showed that dephosphorylation of TYR527 could activate pp60^c-src^ in tumor-derived 4AT and 4BT cell lines [58]. In summary, these bonds all played a key role in protein-compound interaction. In contrast, although several hydrogen bonds and hydrophobic interactions were found in the RELA-palmitic acid pair and SRC-palmitic acid pair, their binding energies were found to be maximal, with the compound-target docking score being -5.0. TP53, AKT1, and MAPK1 not only were the top three targets with the largest degree values but also had high molecular docking scoring values compared with the control group. Based on the points, they are regarded as key targets by which QZC exerts therapeutic effects on GACA. The molecular docking scoring values, coupled with evidence from multiple literatures, indicated that luteolin, rutin, quercetin, and kaempferol were the key active compounds closely related to the treatment of GACA [58–61].

The article "Uncovering the Key Targets and Therapeutic Mechanisms of Qizhen Capsule in Gastric Cancer through Network Pharmacology and Bioinformatic Analyses" was published in 2022. Journal: Comput Math Methods Med.

### 3.8. Survival Analysis

To investigate the prognostic values of the top eight PPI genes, Kaplan-Meier plotter analysis was performed. Analysis results showed that they were not significantly associated with GACA patients' survival. We also found that abnormal expression of these eight PPI genes was not associated with unfavorable RFS or OS in GACA patients either, suggesting that the top eight PPI genes could not be used as biomarkers for GACA (Figure 13).

### 3.9. Data-Based Expression Analysis of PPI Genes as well as Their Corresponding Proteins

TCGA database was used to explore the expression patterns of eight PPI genes (*TP53*, *AKT1*, *EP300*, *HSP90AA1*, *JUN*, *MAPK1*, *RELA*, and *SRC*) in normal and tumor tissues. Results shown in Figure 14(a) indicate that all eight PPI genes were differentially expressed between normal and tumor tissues, with significant differences in the levels of *TP53*, *EP300*, *HSP90AA1*, *JUN*, *RELA*, and *SRC* (*P* < 0.05). Based on clinical characteristics, GACA patients were usually divided into four clinical stages (Stages I-IV). According to the data acquired from TCGA-STAD datasets, correlations between eight PPI gene levels and four clinical stages were analyzed (Figure 14(b)), and results showed that *TP53* and *JUN* genes were significantly associated with clinical stages (Kruskal test, *P* < 0.05). The expression levels of the top eight PPI proteins in normal and tumor tissues were also explored based on the HPA database. As shown in Figure 15, the protein levels of the top eight PPI genes were largely consistent with that of mRNA data.

### 3.10. Inhibition of SGC-7901 Cell Proliferation by Luteolin, Rutin, Quercetin, and Kaempferol

The CCK-8 assay was performed to assess whether or not the predicted four active compounds (luteolin, rutin, quercetin, and kaempferol) could inhibit SGC-7901 cells' proliferation. According to the literature, the tested concentrations of four active compounds were set to 10, 20, 40, 80, and 100 *μ*M for luteolin; 50, 100, 200, 300, and 400 *μ*M for rutin; 10, 20, 40, 80, and 100 *μ*M for quercetin; and 20, 40, 60, 80, and 100 *μ*M for kaempferol. SGC-7901 cells were then treated with four active compounds at the abovementioned concentrations for 48 h. The viability of nontreatment SGC-7901 cells was defined as 100%. The smallest 48 h IC_50_ value was observed in SGC-7901 cells treated by luteolin (36.78), suggesting that luteolin had the strongest inhibitory effect on SGC-7901 cell proliferation among the four, followed by quercetin (62.63), kaempferol (89.59), and rutin (414.4), respectively (Figure 16). Combining with the cytotoxic effects of four compounds on SGC-7901 cells at 24, 48, and 72 h, our data clearly indicated that luteolin, rutin, quercetin, and kaempferol significantly inhibited the proliferation of SGC-7901 cells in a dose- and time-dependent manner.

The article "Uncovering the Key Targets and Therapeutic Mechanisms of Qizhen Capsule in Gastric Cancer through Network Pharmacology and Bioinformatic Analyses" was published in 2022. Journal: Comput Math Methods Med.

### 3.11. Apoptosis of SGC-7901 Cells Induced by Luteolin, Rutin, Quercetin, and Kaempferol

Flow cytometric analysis was carried out to evaluate the apoptosis of SGC-7901 cells induced by luteolin, rutin, quercetin, and kaempferol. Results (Figure 17) demonstrated that, compared to the control group, all four compounds promoted the apoptosis of SGC-7901 cells, with luteolin showing the strongest effect.

### 3.12. Effects of Luteolin, Rutin, Quercetin, and Kaempferol on AKT, P53, and MAPK Protein Levels in SGC-7901 Cells

Three major targets (AKT, P53, and MAPK) predicted by both PPI analysis and molecular docking simulation were further investigated to verify their promotive effects on the apoptosis of SGC-7901 cells through Western blot. As shown in Figure 18, luteolin, rutin, quercetin, and kaempferol significantly decreased levels of AKT, but increased levels of both P53 and MAPK, suggesting that the four compounds inhibited SGC-7901 cell proliferation likely through regulating the signaling pathways related to AKT, P53, and MAPK.

## 4. Discussion

GACA is a common cancer with high mortality [1]. Scientists and doctors have made many efforts in treating GACA patients using a combination of different chemotherapeutic agents. Nevertheless, chemotherapy's efficacy is limited, and the overall 5-year GACA survival rate remains poor (about 27.4%) [62]. It is mainly due to severe adverse effects and multidrug resistance (MDR) in GACA cells that reduce chemosensitivity and efficacy [63]. In contrast, the application of QZC, a Chinese herbal compound, can bypass those side effects and exert a better therapeutic effect. Although the positive effect of QZC in treating GACA has been demonstrated, the mechanisms by which QZC inhibits the proliferation of GACA cells remain unclear. Therefore, to fully develop and better utilize QZC in the future, combined network pharmacology, bioinformatics, and experiments were employed to explore the underlying therapeutic mechanisms of QZC in treating GACA.

The article "Uncovering the Key Targets and Therapeutic Mechanisms of Qizhen Capsule in Gastric Cancer through Network Pharmacology and Bioinformatic Analyses" was published in 2022. Journal: Comput Math Methods Med.

A total of 94 active compounds in QZC and 471 targets were confirmed, which suggested that QZC might treat GACA through multiple targets. Based on the molecular docking simulation results, quercetin, luteolin, kaempferol, and rutin showed high molecular docking values with targets and were anticipated as key active compounds for the anti-GACA effect of QZC. The inhibitory effects of luteolin, rutin, quercetin, and kaempferol on SGC-7901 cell proliferation were verified by the CCK-8 assay, which echoed the molecular docking simulation results. As for quercetin, existing studies have indicated that quercetin can exert its antiproliferation effects by altering cell cycle progression, inhibiting cell proliferation, promoting apoptosis, inhibiting angiogenesis and metastasis progression, and affecting autophagy [64]. In terms of luteolin, it could regulate various signaling pathways (PI3K/AKT and p38 MAPK signaling pathways) to inhibit GACA cell proliferation [65]. Kaempferol has been proven to suppress proliferation and promote autophagy of GACA cells by upregulating miR-181a and inactivating MAPK/ERK and PI3K pathways [66]. Rutin, another pivotal compound identified in this study, exerted its anticancer effect by regulating Wnt/*β*-catenin, P53-independent pathway, PI3K/AKT, JAK/STAT, MAPK, P53, and NF-*κ*B signaling pathways [59]. Therefore, we speculated that QZC, a multicomponent compound, might exert its pharmacological effects in treating GACA through multitargets, which deserves a systematic exploration.

The PPI results demonstrated that TP53, AKT1, EP300, HSP90AA1, JUN, MAPK1, RELA, and SRC were the top eight proteins having more interactions with other protein targets. These eight corresponding genes were subjected to surviving analysis. Of them, *TP53* and *JUN* genes were not only significantly differentially expressed between normal and GACA tissues but also correlated with clinical stages, suggesting that these two genes could serve as underlying biomarkers for GACA patients' prognosis. According to molecular docking simulation results, TP53, MAPK1, and AKT1 that showed a strong affinity with QZC active compounds were considered hub protein targets, and these three hub protein targets were highly likely to interact with QZC active compounds to inhibit GACA cell proliferation. TP53, one of the most frequently mutated genes in human cancer, is a multifunctional transcription factor that induces cell cycle arrest and apoptosis by regulating the expression of its target genes and noncoding genes [67]. Therefore, TP53 is believed to serve as a pivotal regulator that prevents the abnormal proliferation of transformed cells [68]. TP53 has become a hot spot for cancer diagnosis and treatment, and targeting the TP53 oncogenic pathway has become a trend in developing drugs for GACA. Li et al. have mentioned that quercetin increased the expression of TP53 in human GACA. In the present study, we also found an increase in TP53 expression after quercetin treatment, which was consistent with previous studies [61]. MAPK1, a member of the MAPK family, can be targeted and inhibited by miRNAs, resulting in the inhibition of GACA cell proliferation, cell cycle progression, migration, and invasion [69]. Many reports have demonstrated that MAPK1 is an important oncogene that promotes the proliferation, migration, and invasion of GACA cells [70]. It is reasonable to infer that overexpression of MAPK1 is one of the major contributing factors to GACA development. Our study demonstrated that rutin contained in QZC could reduce MAPK1 expression in SGC-7901 cells. In combination with previous studies, rutin might exert antitumor effects against GACA through the MAPK pathway [71]. AKT1 has been shown to promote cell survival and inhibit diverse stimulus-induced apoptosis, including loss of growth factors and cell adhesion [72]. AKT1 is also a potential target for cancer therapy because AKT1 activation is frequently a determinant for tumorigenesis, especially in advanced cancer [73]. Its functions involve activating downstream targets of survival, proliferation, cell cycle regulation, growth, migration, and angiogenesis [48]. In addition, reports have indicated that treating GACA patients with chemotherapy can enhance AKT1 activity, resulting in drug resistance in GACA patients [74]. Therefore, inhibiting AKT1 activity is believed to be an effective way to alleviate drug resistance during chemotherapy [75].

The article "Uncovering the Key Targets and Therapeutic Mechanisms of Qizhen Capsule in Gastric Cancer through Network Pharmacology and Bioinformatic Analyses" was published in 2022. Journal: Comput Math Methods Med.

Abnormal proliferation and insufficient apoptosis in tumor cells are believed to be the two main factors contributing to the onset and development of cancer. Consequently, finding a way to inhibit the proliferation and promote apoptosis of tumor cells would be a potential and effective strategy for cancer treatment. To date, plenty of studies have proved that TCM active compounds fight against cancers by both suppressing tumor cell proliferation and inducing tumor cell apoptosis through diverse signaling pathways [69]. The flow cytometry results confirmed that QZC's four active components (luteolin, rutin, quercetin, and kaempferol) not only inhibited the proliferation of GACA cells but also induced apoptosis of GACA cells.

KEGG pathway analysis showed that genes identified as potential therapeutic targets were enriched in several cancer-related signaling pathways, such as PI3K/AKT signaling pathway, and MAPK signaling pathway. Among them, the PI3K/AKT pathway is often excessively activated in a variety of cancers [76], and several genes that were acquired by PPI analysis in our study belong to the PI3K/AKT pathway. These genes were considered the most available intracellular targets and thus would be ideal for developing small molecular inhibitors. AKT phosphorylation can be intensified due to aberrant activation of the PI3K/AKT pathway [76]. When AKT is phosphorylated, MDM2, one of the major negative regulators of P53, is translocated into the nucleus to ubiquitinated P53, leading to its nuclear exportation and degradation and causing chromosome instability of tumor cells [77, 78]. Aberrantly activating the PI3K/AKT pathway by abnormal expression of these proteins can significantly enhance GACA progression [79]. To verify the predictions of the combined bioinformatic analyses, we performed the Western blotting assay to check the protein levels of AKT, P53, and MAPK in SGC-7901 cells treated with luteolin, rutin, quercetin, or kaempferol, respectively. The results indicated that these four active compounds significantly decreased the protein levels of AKT, but increased the protein levels of both P53 and MAPK. Hence, mediating the pathways containing these targets would be an effective strategy for QZC to exert its anti-GACA effects.

The central idea of TCM has a lot in common with network pharmacology, which is capable of systematically interpreting the treatment process of complicated diseases. In addition to network pharmacology, WGCNA, and data-based gene and protein expression analysis, this study also included molecular experiments to investigate the underlying mechanisms by which QZC exerts effects on GACA at both cellular and molecular levels. Although many advantages are apparent when using the combined approaches, the limitations cannot be neglected. First, a few pivotal targets and active compounds may be ignored if the information from databases was incomplete. Second, various signaling pathways through which QZC exerts its therapeutic effects on GACA were predicted by combined bioinformatic analyses, but experimental verification of the involvement of each pathway was not fully completed. Third, although our results provided important information about the mechanisms by which QZC exerts effects on GACA, further exploration is still needed owning to the complicated therapeutic mechanisms.

The article "Uncovering the Key Targets and Therapeutic Mechanisms of Qizhen Capsule in Gastric Cancer through Network Pharmacology and Bioinformatic Analyses" was published in 2022. Journal: Comput Math Methods Med.

## 5. Conclusion

In summary, luteolin, rutin, quercetin, and kaempferol were identified as the crucial active compounds in QZC. AKT1, MAPK1, and TP53 were predicted to be hub protein targets. Molecular docking simulation suggested that these four active compounds could bind to the three hub protein targets. QZC acts on GACA possibly via regulating multiple signaling pathways, including the MAPK signaling pathway, PI3K/AKT signaling pathway, and TP53 signaling pathway. According to the experimental validation, we believed that QZC exerted therapeutic effects on GACA by regulating the expression of hub target proteins, inhibiting tumor cell proliferation, and enhancing tumor cell apoptosis. Our study elucidated the potential pharmacological mechanisms of QZC in the treatment of GACA and provided new ideas for developing targeted auxiliary anticancer drugs.

## Figures and Tables

**Figure 1:** The technical strategy flowchart for exploring potential mechanisms of QZC against GACA.

**Figure 2:** Analysis of network topology with different soft-thresholding powers.

**Figure 3:** Cluster gene dendrogram with dissimilarity based on topological overlap, together with assigned module colors calculated by WGCNA.

**Figure 4:** Module-trait associations. Each row corresponded to a module eigengene and each column to a trait. Each cell contained the corresponding correlation and *P* value.

**Figure 5:** The drug-compound-target network of QZC. Orange arrows represented herb nodes, green squares represented active compound nodes, and blue circles represented target nodes.

**Figure 6:** Potential targets of QZC in treating GACA. (a) Targets of QZC against GACA in Venn. (b) The PPI network of QZC against GACA. Darker circles represented that these targets had greater correlation degrees with higher degree values.

**Figure 7:** Bar graph of GO enrichment analysis of important genes.

**Figure 8:** Bubble chart of KEGG enrichment analysis of important genes.

**Figure 9:** The network of targets and top 30 pathways. Green squares represented pathways, pink squares represented pathways with high count values, and orange circles represented important targets.

**Figure 10:** The most prominent pathways in GACA. Important targets in pathways were highlighted in pink, and the most relevant targets were highlighted in red. The PI3K/AKT and MAPK signaling pathways were marked in red, enriched significantly, and related to GACA.

The article "Uncovering the Key Targets and Therapeutic Mechanisms of Qizhen Capsule in Gastric Cancer through Network Pharmacology and Bioinformatic Analyses" was published in 2022. Journal: Comput Math Methods Med.

**Figure 11:** The heat map of 72 compound-target docking scores. Darker color represented lower molecular docking score. Pro-lig was used as the control.

**Figure 12:** The sketch map of ten compound-target pairs: (a) MAPK1-luteolin, (b) SRC-luteolin, (c) EP300-rutin, (d) AKT1-rutin, (e) SRC-rutin, (f) HSP-rutin, (g) TP53-rutin, (h) MAPK1-que, (i) SRC-quercetin, and (j) SRC-kaempferol.

**Figure 13:** Kaplan-Meier curves of top eight PPI genes in GACA: (a) TP53, (b) EP300, (c) AKT1, (d) MAPK1, (e) SRC, (f) RELA, (g) JUN, and (h) HSP90AA1.

**Figure 14:** The mRNA expression levels of the top eight PPI genes in GACA patients: (a) mRNA expression levels between normal and GACA tissues; (b) mRNA expression levels in four clinical stages (Stages I-IV).

**Figure 15:** Protein expression levels of TP53, EP300, AKT1, MAPK1, SRC, RELA, JUN, and HSP90AA1 in normal and GACA tissues based on immunohistochemistry data from HPA.

**Figure 16:** Inhibitory effects of four active compounds on SGC-7901 cells' proliferation: (a) quercetin; (b) kaempferol; (c) luteolin; (d) rutin; (e) time-dependent inhibitory effects of four active compounds on SGC-7901 cells' proliferation. The data were expressed as mean ± SD (*n* = 3).

**Figure 17:** Apoptosis of SGC-7901 cells treated with four active compounds for 24 h: (a) control, (b) quercetin, (c) rutin, (d) kaempferol, and (e) luteolin.

**Figure 18:** Effects of four active compounds on protein levels of p-AKT, AKT, p-P53, P53, p-MAPK, and MAPK in SGC-7901 cells: (a) control, (b) quercetin, (c) rutin, (d) kaempferol, and (e) luteolin. ^∗^*P* < 0.05, ^∗∗^*P* < 0.01, and ^∗∗∗^*P* < 0.001 vs. control group.

**Table 1:** Compounds collected through the literature and their network parameters.

Mol ID	Compound	PubChem CID	OB (%)	DL	Herb
MOL000114	Vanillic acid	8468	35.47	0.04	AR
MOL000415	Rutin	5280805	3.2	0.68	AR; PR
MOL000098	Quercetin	5280343	46.43	0.28	AR; NRER; PR
MOL000069	Palmitic acid	985	19.3	0.1	AR; NRER; IF
MOL000391	Ononin	442813	11.52	0.78	AR
MOL000421	Nicotinic acid	938	47.65	0.02	AR; IF
MOL000412	Mucronulatol	442811	4.22	0.26	AR
MOL000211	Mairin	64971	55.38	0.78	AR
MOL000356	Lupeol	259846	12.12	0.78	AR; PR
MOL000131	Alpha-linoleic acid	5280450	41.9	0.14	AR
MOL000416	Lariciresinol	332427	5.53	0.38	AR
MOL000422	Kaempferol	5280863	41.88	0.24	AR; PR
MOL000239	Jaranol	5318869	50.83	0.29	AR
MOL000354	Isorhamnetin	5281654	49.6	0.31	AR
MOL000439	Isomucronulatol 7,2′-di-O-glucoside	15689653	49.28	0.62	AR
MOL005928	Isoferulic acid	736186	50.83	0.06	AR
MOL000437	Hirsutrin	5280804	1.86	0.77	AR
MOL000296	Hederagenin	73299	36.91	0.75	AR
MOL000388	Gamma-aminobutyric acid	199	24.09	0.01	AR
MOL000392	Formononetin	5280378	69.67	0.21	AR
MOL000389	Ferulic acid	1548883	54.97	0.06	AR
MOL000433	Folic acid	6037	68.96	0.71	AR; MAR
MOL000390	Daidzein	5281708	19.44	0.19	AR
MOL000431	Coumarin	323	29.17	0.04	AR
MOL000417	Calycosin	5280448	47.75	0.24	AR
MOL000387	Bifendate	108213	31.1	0.67	AR
MOL000430	Betaine	247	40.92	0.01	AR
MOL000411	Astraisoflavanin	131420	18.37	0.86	AR
MOL000378	7-O-Methylisomucronulatol	15689652	74.69	0.3	AR
MOL000418	Calycosin 7-O-glucoside	5318267	10.05	0.81	AR
MOL000371	3,9,10-Trimethoxypterocarpan	15689655	53.74	0.48	AR
MOL000442	1,7-Dihydroxy-3,9-dimethoxy pterocarpene	5316760	39.05	0.48	AR
MOL000432	Linolenic acid	5280934	45.01	0.15	AR
MOL000380	Astrapterocarpan	14077830	64.26	0.42	AR
MOL000396	(+)-Syringaresinol	443023	3.29	0.72	AR
MOL001494	Mandenol	5282184	42	0.19	NRER
MOL001792	Liquiritigenin	114829	32.76	0.18	NRER
MOL002879	Diisooctyl phthalate	33934	43.59	0.39	NRER
MOL000449	Stigmasterol	5280794	43.83	0.76	NRER
MOL005344	Ginsenoside Rh2	119307	36.32	0.56	NRER
MOL002153	Spathulenol	92231	82.33	0.12	NRER
MOL000252	Farnesol	445070	28.44	0.06	NRER
MOL000263	Oleanolic acid	10494	29.02	0.76	NRER
MOL002818	4′-Hydroxyacetophenone	7469	36.8	0.03	NRER
MOL002850	Butylated hydroxytoluene	31404	40.02	0.07	NRER
MOL000305	Lauric acid	3893	23.59	0.04	NRER
MOL000908	Beta-elemene	6918391	25.63	0.06	NRER
MOL000675	Oleic acid	445639	33.13	0.14	NRER
MOL007500	Panaxatriol	73599	15.42	0.79	NRER
MOL007501	Panaxydol	126312	61.67	0.13	NRER
MOL000879	Methyl palmitate	8181	18.09	0.12	NRER
MOL001863	Methyl 14-methylpentadecanoate	21205	9.42	0.11	NRER
MOL000384	DL-Glucuronic acid	65041	3.35	0.04	NRER
MOL005285	(20S)-Protopanaxadiol	11213350	29.69	0.77	NRER
MOL005338	Ginsenoside Re	441921	4.27	0.12	NRER
MOL012662	Ginsenoside F1	9809542	4.05	0.61	NRER
MOL005331	Ginsenoside rb1	9898279	6.24	0.04	NRER
MOL005333	Ginsenoside Rb2	6917976	6.02	0.04	NRER
MOL007479	Ginsenoside Rc	12855889	8.13	0.04	NRER
MOL011400	Ginsenoside Rf	441922	17.74	0.24	NRER
MOL012332	Ginsenoside RG2	21599924	8.32	0.25	NRER
MOL012334	Ginsenoside Rg3	9918693	12.43	0.22	NRER
MOL011407	20(S)-Ginsenoside Rh1	12855920	8.4	0.57	NRER
MOL005325	Ginsenoside Ro	11815492	1.98	0.05	NRER
MOL009956	Gypenoside XVII	44584555	3.51	0.1	NRER
MOL013377	Lutein	5281243	22.59	0.55	NRER
MOL001771	Clionasterol	457801	36.91	0.75	IF
MOL001781	Indigo	10215	38.2	0.26	IF
MOL001810	Qingdainone	3035728	45.28	0.89	IF
MOL002309	Indirubin	10177	48.59	0.26	IF
MOL002311	Glycyrol	5320083	90.78	0.67	IF
MOL002318	C05837	6602378	66.02	0.48	IF
MOL002322	Isovitexin	162350	31.29	0.72	IF
MOL001456	Citric acid	19782904	56.22	0.05	IF
MOL001766	5-Hydroxyoxindole	76955	59.16	0.04	IF
MOL001801	Salicylic acid	338	32.13	0.03	IF
MOL001808	Tryptanthrin	73549	19.28	0.29	IF
MOL000346	Succinic acid	21952380	29.62	0.01	IF
MOL000635	Vanillin	1183	52	0.03	IF
MOL000140	Diosgenin	99474	12.67	0.82	PR
MOL005241	Pennogenin	12314056	16.93	0.78	PR
MOL004718	Alpha-spinasterol	5281331	42.98	0.76	PR
MOL001987	Beta-sitosterol	222284	33.94	0.7	PR; NRER; IF
MOL006096	Isorhamnetin-3-O-neohesperidoside	11664505	4.45	0.68	PR
MOL000006	Luteolin	5280445	36.16	36.16	PR
MOL004368	Hyperoside	5281643	6.94	0.77	PR
MOL000676	Dibutyl phthalate	3026	64.54	0.13	PR
MOL009295	Flazin	5377686	94.28	0.39	PR
MOL002441	Dioscin	119245	17.75	0.06	PR
MOL008320	Ecdysterone	5459840	6.94	0.82	PR
MOL007751	Ajugasterone C	441826	5.31	0.81	PR
MOL003887	Gracillin	159861	27.39	0.06	PR
MOL003971	Threonin	6288	73.52	0.01	MAR
MOL002223	Tau	4068592	24.37	0.01	MAR

The article "Uncovering the Key Targets and Therapeutic Mechanisms of Qizhen Capsule in Gastric Cancer through Network Pharmacology and Bioinformatic Analyses" was published in 2022. Journal: Comput Math Methods Med.

## Data Availability

The data used to support the findings of this study are available from the corresponding author upon request.
